This article has been retracted.

# Prevalence of active trachoma infection and associated factors post‐war resettled population in raya kobo districts, North East Ethiopia: A community‐based cross‐sectional study in 2022

**DOI:** 10.1002/hsr2.1486

**Published:** 2023-08-06

**Authors:** Fassikaw Kebede, Muhammad Jamal

**Affiliations:** ^1^ Department of Epidemiology and Biostatics College of Health Science Woldia University Woldia Ethiopia; ^2^ Mersa Health Centre Habru Woreda North Wollo North Wollo Ethiopia

**Keywords:** active trachoma, displaced population, Ethiopia

## Abstract

**Background:**

Active trachoma infection poses a serious threat to public health, particularly for those who live in an unprivileged area and has practiced open‐field defecation. This study aimed to estimate the prevalence of active trachoma infection and associated factors in the post‐war resettled population in Raya Kobo district, North East Ethiopia: a community‐based cross‐sectional study in 2022.

**Methods:**

A community‐based cross‐sectional study was conducted among 602 participants randomly selected in 14 slum villages in Raya Kobo from February 16th to March 30th, 2023. After the data was collected using a semi‐structured questionnaire and entered into Epi‐data version 3.2. The study participants were chosen using a two‐stage sampling process. Binary logistic regression was used to identify factors for active trachoma infection. Adjusted odds ratios (AORs) with 95% confidence intervals (CIs) were claimed for the strength of association at *p* < 0.05.

**Results:**

Overall, 602 (99.9%) study participants were included in the final analysis. At the end of the study period, 126 (20.9) participants developed active trachoma infection. On multivariable analysis, were aged ≥45 years (AOR = 7.9, 95% CI = 2.4–25.3), history of eye infection (AOR = 3.7, 95% CI = 2.4–10.4, *p* = 0.001), were poor wealth index (AOR = 9.2, 95% CI = 2.7–23.7), having separated kitchen (AOR = 4.05, 95% CI = 1.86–8.86), living with animals (AOR = 5.92, 95% CI = 2.31–14.7) and having got administration of mass‐drug (AOR = 8.9, 95% CI = 2.36–33.6) were significant risk factors for active trachoma infection. Whereas, face washing practice regularly (AOR = 0.23, 95% CI = 0.127–0.43), and toilet availability (AOR = 0.35, 95% CI = 0.20–0.97) were preventive factors for active trachoma infection.

**Conclusion:**

A significant prevalence of active trachoma infection was reported in the area as compared with previous findings and urgent clinical intervention, and the WHO critical SAFE strategies (surgery, antibiotics, facial cleanliness, and environmental improvement) implementation is highly needed in the area. In addition, healthcare providers should focus on information dissemination on proper latrine utilization, and washing the face regularly to prevent active trachoma infection is highly recommended.

## 1 INTRODUCTION

Chlamydia trachomatis is an infectious eye disease caused by *Chlamydia trachomatis*, an obligate intracellular bacterium that causes follicular conjunctivitis, superficial keratitis, and corneal and finally caused scarring.^1^, ^2^ Active trachoma infection is characterized by severe corneal abrasion, increased inflammation, and scarring of tarsal conjunctivitis due to insufficient secretion of biomarkers for ocular diseases and neurodegenerative condition of eyes.^3^, ^4^ Pathologically, persistent and recurrent eye infections cause inflammation of the outer cornea and ocular surface, which fails to connect the sensory and motor nerves for correct imaging of the eyes.^5^, ^6^

Globally, active trachoma is the leading infectious cause of blindness and is considered the cause of visual impairment in 1.9 million people.^7^, ^8^ Around 50 million individuals worldwide have trachoma, and 3–10 million of them go blind as a result of the infection^9^ with annual economic lost $2.9 and $5.3 billion.^9^, ^10^ According to the World Health Organization (WHO) 2020, more than 88% of the 157.7 million people living in the area with active trachoma sites were from African countries with more than 44.2%.^11^, ^12^

The WHO promotes a multifaceted “SAFE” method for trachoma prevention, which includes multiple components for reducing the burden through antibiotic distribution and environmental sanitation, and in 2021 achieved antibiotic coverage of 44%.^12^, ^13^ A 10% post‐surgery relapse was reported despite this success with more than 80% chemo‐prophylaxis coverage and 47.6% surgical intervention in highly active trachoma mapping zones.^14^, ^15^ However, in Ethiopia, the combined prevalence of active trachoma was found to be 26.9% in school‐age children and 4.1% in the adult population, according to recent meta‐analysis findings^16^, ^17^ and the problem is exacerbated by a lack of clean water, living in in a health center, and family size.^6^, ^18^

More than 1.4 million people were forced to reside in refugee camps during the battle against the Tigray People Liberation Front (TPLF) and the central government of Ethiopia, particularly the frontline of the war of Amhara and Afar areas, where 600,000 people died.^19^ As a result, the community was forced to move, which made them more vulnerable to communicable diseases including active trachoma, infection, food insecurity, and subpar medical care. Therefore, our study aimed to estimate the post‐war burden of active trachoma among the displaced population in Raya Kobo District in North Wollo Zone, North East Ethiopia.

### 1.1 Methods and study setting

This study was conducted in Raya Kobo Woreda, located in Amhara Region. which is located 552 and 365 km from the regional capital city Bahir Dare and Addis Ababa, respectively.^20^ The Amhara region, more specifically the North Wollo zone, has already lost more than 2347 healthcare facilities that give service to the catchment population.

### 1.2 Study design and period

The community‐based cross‐sectional study was employed among randomly selected 14 displaced slums/shantytowns in Raya Kobo district, North East Ethiopia.

### 1.3 Study population

All individuals who reside from February 16th to March 30th, 2023 among randomly selected residents in Raya Kobo District post‐war on TPLF.

#### 1.3.1 Inclusion criteria

All individuals who had lived in Raya Kobo district post‐war randomly selected households were interviewed for at least a month and included in this study.

### 1.4 Sample size determination

The sample size was calculated using a single proportion formula since there is no research about TT infection post‐war in northern Ethiopia about TT infection with considering the following parameters and the formula of the single population proportion

*N* = *Z*@/_2_*p (*p* − *q*)/*d* ^2^*

*Z* = 1.96 (95% confidence interval)

*p* = 0.5% (assumption)

*d* = 0.05, merging error

*n* = 3.84*0.5 (0.5)/0.0025, and considering,

*d* = design effect; 1.5 since the study used multistage sampling, nonresponse rate =5%. The final sample size was 602.4; we interviewed 602 participants from 602 households.

### 1.5 Sampling techniques and procedure

A multistage sampling process was used to ensure the representation of all residents in the Raya Kobo district to select the study population. First, 14 refuge slums or administrative (villages) were randomly selected by lottery method from the total 45 districts. Second, the proportional sampling technique was accompanied for each administrative slum based on their baseline population distribution which is available and taken from Woreda administrative. Then we determined the sampling fraction (*K*) for the selection of each administrative site based on the value which is given in the formula

$$\begin{array}{l} K=\frac{\text{Total household in kebele}}{\text{Final sample size}}=8762/602=12\;\\ \;\; \end{array}$$

We selected 602 people for the interview after a proportional sample was given for each of the 14 administrative villages. The researchers chose 602 individuals using a random sampling procedure, which involved first writing down their names on a sheet of paper, choosing one family by lottery, and then asking questions in the participants' native tongue.

### 1.6 Study variables

#### 1.6.1 Dependent variable

Trachoma presence (yes/no)

#### 1.6.2 Independent variables

1. These included age, sex, religion, wealth index, number of children, family size, occupation, face washing practice, frequency of face washing, educational status, smoking, and drinking behaviors, face washing frequency, history of epilation, history of annual Zithromax, information about trachoma, utilization of soap for face, Repeated eye infection, availability of toilets, residence, distance to the health care center, distance to get water, distance to health facilities, solid waste disposal, and liquid waste disposal, having a kitchen in the living room, and living with a domestic animal were considered independent variables.

### 1.7 Operational definition

#### 1.7.1 Active trachoma

The diagnosis of active trachoma was accompanied by two clinicians, both by a history taken from the respondents and following rapid examination followed by two medical to detect active trachoma infection if the cases are suspected binocular magnifying loupes (×2.5) was used for confirmation.^12^, ^21^

### 1.8 Data collection tools

Before data were collected to increase the identification and referral system of active trachoma cases during data collection, a novel approach using standard screening questions and a card was used to identify active trachoma. For confirmation purposes, data collectors selected two medical doctors' holders with Integrated Eye Care Workers, which helps to confirm the diagnosed and easily graded trachoma. Data were collected using a pretested and interviewer‐administered structured questionnaire which was adapted from different literature on cross‐sectional survey research.^22^, ^23^, ^24^

### 1.9 Data quality assurance

The quality of data was ensured at the point of data collection and data entry. Emphasis was given to designing questionnaires on the objective of the study and explained to data collectors. A pretest was undertaken on 5%^25^ of our final samples at the Habru site with the prepared structured questionnaire before the actual data collection started and the amendment was made to the format.

### 1.10 Data processing and analysis

The collected data were entered and cleaned using Epi Info software version 7, and then exported to STATA (SE) R/14) data for further analysis. Frequency and percent were computed through bivariable analysis to obtain summary statics. Bi‐variable analysis between the dependent and independent variables was performed separately using logistic regression. In addition, a chi‐square analysis was performed for each variable to assess whether statistical significance was reported among categorical variables. The strength of association between dependent variables and independent variables is expressed as an adjusted odds ratio (OR) within 95% confidence interval (CI).

## 2 RESULTS

### 2.1 Socio‐demographic characteristics of participants

Six‐hundred‐two (602) participants were included with an overall response rate of 100%. The majority, 361 (60%) of the participants were females and nearly half of 300 (49.8%) of them were within 30–44 years of age. More than half, 320 (53.2%) of the interviewees had no formal education; however, 19.6% of the participants had completed high school. The largest proportion, 437 (72.6%) of the study participants were farmers and 418 (69.4%) of them were rural dwellers, see Table 1.

**Table 1:** Baseline socioeconomic and environmental characteristics of respondents with active trachoma burden in Raya Kobo district from February 16th to March 30th, 2023.

Variable	Category	Frequency	Percent (%)
sex	Male	241	40.0
	Female	361	60.0
Age	≤30	204	33.9
	30–44	300	49.8
	≥45	98	16.3
Marital status	Single	115	19.1
	Married	393	65.3
	Divorced	94	15.6
Responsibility	Head	469	77.9
	Family member	133	22.1
Number of children in the house	No children	27	4.49
	One	421	69.9
	≥Two	154	25.6
Occupation status	Farmer	437	72.6
	Merchant	99	16.4
	Employer	21	3.5
	Other	45	7.5
Educational status	No formal education	328	53.2
	Complete junior	162	27.1
	High school and above	112	19.8
Residence	Urban	184	30.6
	Rural	418	69.4
Religious	Orthodox	384	63.8
	Muslim	163	27.1
	Protestant	43	7.1
	Catholic	12	2.0
Wealth index	Poor	201	33.3
	Medium	200	33.3
	Rich	201	33.3
Washing face per day	Once	97	16.1
	Twice	231	38.4
	More than three	274	45.5
Using soap	Yes	487	80.9
	No	115	19.1
Available of Toilet	Yes	385	64.1
	No	217	35.9
Time to water source	≥30 min	506	84.1
	≤30 min	96	15.9
Distance to a health facility	<10 km	508	84.9
	≥10 km	98	15.9
Had Waste disposal	Yes	500	83.1
	No	102	16.9
Domestic animals	Yes	212	35.2
	No	390	64.8
Separated kitchen	Yes	501	83.2
	No	101	16.8
water source types	Pipe	284	47.2
	Well	171	28.4
	Pond	81	13.5
	River	66	11.1
Information about trachoma	Yes	561	93.9
	No	41	6.8
Information about trichiasis	Yes	534	88.7
	No	68	11.3
TT can cause blindness	Yes	497	82.6
	No	105	17.4

### 2.2 Behavioral characteristics of respondents

The largest proportion of 561 (93.9%) of the respondents had information about trachoma infection. More than half of the 385 (64.1%) studies sampled had latrines but not 217 (35.9%). The largest proportion of 500 (81.5%) of the study participants had disposal (either solid or liquid) nearby their household, but 212 (35.2%) lived with animals. More than half of the (63.5%) sampled population were orthodox believers, and 274 (45.5%) of them regularly washed their faces, see Table 1.

### 2.3 History of eye infection

Of the 602 participants in total, 58 (or 9.6%) had a history of eye infection, and 42 (or 7.1%) of those had recurrent infections. However, 13 (6.3%) and 18 (3%), respectively, of the responders had undergone TT surgery and had previously experienced ocular epilation (Relapse). Azitromaxine chemoprophylaxis was administered in large doses to more than half of the research participants (Table 2).

**Table 2:** Medical‐related characteristics of the post‐war burden of TT infection among people living in Raya Kobo District, North East Ethiopia.

Variables	Category	Frequency	Percent (%)
History of eye infection (*N* = 602)	Yes	58	9.6
	No	544	90.4
History of epilation (*N* = 602)	Yes	18	3.0
	No	584	97
History of TT surgery (*n* = 13)	Yes	13	6.3
	No	589	93.7
Active trachoma infection (*N* = 602)	Yes	126	20.93
	No	476	79.07
Tricuris tricuarias TT infection (*N* = 602)	Yes	98	16.3
	No	504	83.7
Site of TT infection (*n* = 98)	Right	19	19.4
	Left	45	45.9
	Both	34	34.7
Mass drug administration	Yes	527	87.5
	No	75	12.5

### 2.4 Burden and grading of active trachoma infection

At the end of the study period, 126 (20.93%) of them confirmed active trachoma infection and 94 (15.6%) of those were stage IV trachoma infection. More than one fourth, 34 (26.9%) of the respondents had age ≤30 years and 47 (37.3%) were a poor class of wealth index. The majority, 94 (74.6%) of the cases were TT infection (stage IV), while the remaining 16 (12.76%), 8 (6.3%), 6 (4.7%), and 3 (2.5%) were found to be stage I, stage II, stage III, and stage IV active trachoma infections, respectively, see (Figure 1.

**Figure 1:** Active Trachoma Stage among Diagnosed Population in Raya Kobo District.

### 2.5 Factors associated with active trachoma infection

During the bivariable logistic regression, factors including age, sex, residence, marital status, occupation status, wealth index, number of families living with animals, face washing practice, information about trachoma, history of mass drug administration, separated kitchen from the living house, history of eye infection, availability of toilets, distance to the health care center, and time to get drinking water were a candidate for multivariable regression at *p* ≤ 0.25 using forward selection and backward elimination.

After controlling certain confounding during multivariable regression, variables including age≥45 years, poor wealth index, face washing practice, distance to get drinking water, history of previous eye infection, mass drug administration, toilet, and history of eye infection were associated with active trachoma infection.

Accordingly, when the respondents aged≥45 years were 7.9 (AOR = 7.9(2.4‐ 25.3, *p* = 0.001) times increased odds of active trachoma infection as compared to those aged <30 years.

Likewise, respondents with a history of eye infection per year were 3.7 (AOR = 3.7: 95%CI: 2.4‐ 10.4, *p* = 0.001) time increased the odds of active trachoma infection as compared with the counter group.

Compared to the rich wealth index group of respondents, being poor in an economic class of the displaced population had 9.2(AOR = 9.2, 95%CI: 2.7, 23.7, P = 0013) times increased odds of developing active trachoma infection.

Similarly, an individual who washed and had practiced face washing regularly were 77% reduced odds of developing active trachoma infection as compared with the counter group (AOR = 0.23, 95%CI;0.127‐‐0.43)*.

The log odds of active trachoma infection developing was 65% (AOR = 0.35, 95%CI: 0.20‐ 0.97, *p* = 0.013) time reduced for having a toilet in their household in contrast with no toilet household.

Likewise, the log odds of active trachoma infection were four (AOR = 4.05; 95%CI: 1.86‐‐ 8.86, *p* = 0.001) times increased for participants and those who had no separated Kitchen from the main house as compared with the counter group.

Finally, participants had no history of mass drug chemoprophylaxis (Zithromax) for prevention of active trachoma 8.9(AOR = 8.9:95%; 2.36‐‐33.6, *p* = 0.01) time increased to develop active trachoma infection as compared with counter groups see **(**Table 3 **)**.

**Table 3:** Bi‐variable and multivariable logistic regression to identify factors associated with active trachoma infection among the resettled population in Raya Kobo District, Northeast Ethiopia.

Variables	Categories	Active trachoma		COR (95% CI)	P= value	AOR (95% CI)
		Yes	No			
**Sex**	Male	35	204	Ref		Ref
	Female	91	272	1.97(1.26–2.99)	0.002	2.29(0.56–9.31)
**Age**	≤30	30	174	Ref		Ref
	30‐44	47	253	1.07 (0.65–1.77)	0.76	1.28(0.43–3.27)
	≥45	49	49	5.81(3.3–10.1)	0.017	7.9(2.41–25.30)*
**Resident**	Urban	19	165	Ref		Ref
	Rural	107	311	2.98(1.77–5.04)	0.011	1.99(0.56–9.**1)**
**Marital status**	Single	8	107	Ref		Ref
	Married	91	302	1.63(0.98–8.95)	0.025	1.3(0.39–4.28)
	Divorce/widowed	27	67	1.42(1.35‐5.74)	0.019	0.85 (0.18–3.97)
**Occupation status**	Farmer	105	336	2.0(1.71–3.22)	0.018	0.43(0.11–1.69)
	Merchant	11	83	2.51(0.87–7.21)	0.213	0.301(0.11–2.31)
	employer	4	20	1.77(0.99–4.34)	0.241	
	Students	6	36	Ref		Ref
**Wealth index**	Poor	52	66	**4.47(2.79–12.39)**	**0.001**	2.9 (1.09–7.17)*
	Medium	43	184	2.7(0.93–3.45)	0.159	1.6(0.59–5.61)
	Rich	31	226	Ref		Ref
**Family members**	No	2	25	Ref		Ref
	One	46	375	1.61(0.35–6.62)	0.59	1.12(0.162–7.475)
	≥2	78	76	12.8 (1.92–56.07)	0.002	1.6(0.22–11.78)
**Living with animal**	Yes	89	47	3.79 (2.3–6.17)	0.001	1.2(0.39–11.7)
	No	37	429	Ref		Ref
**Face washing practice**	Not at all/day	62	35	Ref		Ref
	At least once/a day	21	210	0.17 (0.3–0.85)	0.001	0.87(0.13, 1.29)
	More than two	43	231	0.11(0.062–0.177)	0.001	0.23(0.127–0.43)*
**Information about trachoma**	Yes	87	474	Ref		Ref
	No	39	2	68(28.6–165.9)	0.001	3.1(0.36–33.6)
**History of Eye infection**	Yes	52	6	28.2(21.5–69)	0.001	3.46(2.37–16.4)*
	No	74	474	Ref		Ref
**Time to get water**	<30 min	41	416	Ref		Ref
	≥30 min	85	16	8.7 (4.99–39.3)	0.069	1.02(0.93–11.31)
**Health facility distance**	< 10 km	47	459	1.9(0.5–3.6)	0.78	1.93(0.53–3.60)
	≥10 km	79	17	Ref		Ref
**Toilet availability**	Yes	59	326	0.45(0.27–0.604)	0.023	0.35(0.20–0.97)*
	No	67	150	Ref		Ref
Mass drug administration (MDA)	No	59	6	38(28.6–65.9)	0.001	8.9(2.36–33.6)*
	Yes	67	470	Ref		Ref
**Having waste disposal**	Yes	49	451	Ref		Ref
	No	77	25	28.3(16.5–48.5)	0.001	23.93 (11.15–51.3)*
**Separated kitchen**	Yes	41	460	Ref		Ref
	No	85	16	59.6(31.9–111.06)	0.001	4.05(1.86–8.86)*

## 3 DISCUSSION

In Ethiopia, trachoma is the leading infectious disease that causes blindness.^7^ At the end of this study, 126 (20.93%) participants were developing active trachoma infections. This makes the overall active trachoma infection post‐war among the resettled population in Raya Kobo District found to be 20.93% (95%CI: 17.85‐‐‐24.37). This report is high than compared to previous finding 6% in Dangilla,^7^ 11.8% in Metema,^26^ and 6.65% in Brazil.^27^ The major reason for the discrepancy may be our study report was compiled post‐war among displaced and resettled populations, which may increase the estimation in addition to differences in the sample size and environmental characteristics of the comparison groups.

Conversely, the final report of our study is also most consistent with previous findings with 17.2% in Gambella,^28^ 18% in Dembia,^29^ 18.6% in Dera Woreda,^30^ 17.5% in Howassa,^11^ and 17.5% in Sudan.^11^ Whereas, our study finding is lower than 23.4% reported in Oromia,^23^ 26.9% meta‐analysis in Ethiopia,^16^ 37.9%in Wolyita,^31^ and 58.5% in Wagehemra Zone.^25^ This may be due to the difference in socioeconomic, demographic, and geographical variation among the included study populations. As indicated by the fact that 385 (63.95%) of the population had standard latrines, the presence of latrines among the population who had been resettled had significantly improved during data collection to attain zero open defecation cases reported after the conflict in districts.

Regarding associated factors with active trauma, age ≥45 years for study participants was 7.9 (AOR = 7.9(2.4‐ 25.3, *p* = 0.001) times increased odds of developing active trachoma infection as compared with age <30 years. This finding is consistent with the previous study reported in Shewa,^6^ Tigray, Southern Sudan,^15^, ^32^, ^33^ and Colombia.^34^ This might be because when age gets older; the immune response may decrease and one can be exposed easily to different communicable infections. In some instants, when age is increased, lacking the habit of frequent face washing and considered considering that the non‐use of soap can increase the probability of having active trachoma [19], and there are difficulties for older age than childhood age to apply permanently. Moreover, it can when age increases, there seems to be a challenge in implementing the SAFE strategy's “F“ component, and there is also a tendency to forget about active trachoma infections due to a lack of awareness of the possibility that increased nasal and ocular discharge will result in an increased risk of transmission.

In a multivariable analysis of this study, individuals who practice regularly washed face were 77% (AOR = 0.23, 95%CI; 0.127‐‐0.43) times preventing the likely hood of getting active trachoma infection as compared with the counter group. This is consistent with findings reported in Awi‐Zone, Southwest Ethiopia,^35^, ^36^ Howassa City,^11^ and South Sudan.^37^ This might be significantly associated with the fact that an unclean face could be more likely to spread ocular secretions infected with C. trachomatis and highly susceptible to the risk of developing.^15^

In this study, we found that having access to latrine use reduces the risk of active trachoma infection by 65% (AOR = 0.35, 95%CI: 0.20‐ 0.97, *p* = 0.013) when compared to people without latrines. This is consistent with the previous finding in Oromia, Burundi,^38^, ^39^ wilayat^15^ Dera,^30^ and Metema.^26^ This could be due to the presence of open file deification of feces as a breeding medium for the trachoma fly vector ***Musca sorbent*** which leads to a higher chance of transmission of active trachoma infection from the person who didn't have a toilet in their household.

In the final report of our study, the odds of having active trachoma infection among study participants with those who had repeated eye infections were threefold increased as compared with no history of eye (AOR = 3.7: 95%CI: 2.4‐ 10.4, *p* = 0.001). Consistent with earlier research findings,^3^ cleaning one's face with soap and water has proved crucial in reducing the occurrence of many eyes and associated infections, especially in children.

This study investigated ‘the poor wealth index class of respondents was 9.2 (AOR = 9.2, 95%CI: 2.7, 23.7, P = 0013) times increasing the odds of developing active trachoma infection as compared with the rich economic class and this was consistent with the previous finding in Dangila woreda.^7^ The main reason for this similarity might be that active trachoma infection is almost exclusively a disease for poor families and communities, and those who lead a destitute life including orphaned and old age people are highly susceptible to active trachoma infection

This is consistent with the previous finding in Malawi ^40^ that the log odds of active trachoma infection was four (AOR = 4.05; 95%CI: 1.86‐‐ 8.86, *p* = 0.001) increased for participants who had no separated kitchen from the main house as compared with the counter group had separated kitchen. This could be caused by the clustering of infections in the home structure and inside the kitchen in a household, which is regarded to be a significant trait of trachoma infection and an essential epidemiological aspect of many infectious diseases including trachoma infection.^41^

In this report, there was an 8.9(AOR = 8.9:95%; 2.36‐‐33.6, *p* = 0.01) time increase for active trachoma infection if mass drug administration of Azitromza as part of chemoprophylaxis for prevention. A recent Cochrane review of four cluster randomized trials (RCTs) that compared community‐level treatment with MDA‐azithromycin showed a reduction of 40–60% active trachoma within 12 months of treatment as compared with control groups supporting the use of MDA‐azithromycin in trachoma control as being highly acceptable.^42^, ^43^

Unlike previous studies, finding in central Ethiopia,^44^ Southern Ethiopia,^45^ and Tanzania^46^ demonstrated that our study had no evidence of distance to drinking water sources, distance to health facilities, and many families and no significant association with acquiring to develop active trachoma infection. Individuals who lived near water sources had higher hygiene standards, more personal cleanses, and a lower risk of trachoma infection from flies, which is directly related to the likelihood of developing Trachoma.^47^

### 3.1 Limitations of the study

The study may be prone to reporting bias since some of the data was collected based on self‐reported information and this study did not use the qualitative method to explore other factors contributing to the final results

## 4 CONCLUSION

A significant prevalence of active trachoma infection was reported in the area as compared with previous findings and urgent clinical intervention and the WHO critical SAFE strategies (surgery, antibiotics, facial cleanliness, and environmental improvement) implementation is highly needed in the area. In addition, the health care provider should focus on information dissemination on proper latrine utilization, and washing the face regularly to prevent active trachoma infection is highly recommended.

## AUTHOR CONTRIBUTIONS

**Fassikaw Kebede**: Conceptualization; data curation; formal analysis; funding acquisition; investigation; methodology; project administration; resources; software; supervision; validation; visualization; writing—original draft; writing—review and editing. **Muhammad Jamal**: Conceptualization; data curation; formal analysis; funding acquisition; investigation; methodology; project administration; visualization; writing—original draft; writing—review and editing.

## CONFLICT OF INTEREST STATEMENT

The authors declare no conflict of interest.

## ETHICS STATEMENT

The study was carried out under the Helsinki Declaration and the ethical review board of Woldia university college of Health Science Research And Community Service, Technology‐Transformation, And University‐Industry Linkage office ethically cleared this research to conduct refill number (RCS, TT & UIL; 0015/2015) on 09/02/2015 E.C. written informed consent was obtained from each participant during data collection.

## TRANSPARENCY STATEMENT

The lead author Fassikaw Kebede affirms that this manuscript is an honest, accurate, and transparent account of the study being reported; that no important aspects of the study have been omitted; and that any discrepancies from the study as planned (and, if relevant, registered) have been explained.

## Supporting information

Supporting information.

## Data Availability

The data set analyzed for this study is from the corresponding author on reasonable request.
